This article has been retracted.

# Robust Transmit Beamforming Algorithm for Low-Altitude Slow-Speed Small Target Detection

**DOI:** 10.1155/2022/6358133

**Published:** 2022-06-08

**Authors:** Songpo Jin, Hongtao Li, Pengyi Wang, Yi Shen, Shanna Zhuang

**Affiliations:** ^1^The 54th Research Institute of China Electronics Technology Group Corporation, Shijiazhuang 050081, China; ^2^School of Electronic and Optical Engineering, Nanjing University of Science and Technology, Nanjing 210094, China; ^3^School of Information and Science Technology, Shijiazhuang Tiedao University, Shijiazhuang 050043, China

## Abstract

Strong ground clutter echoes make it difficult to detect low-altitude slow-speed small (LSS) targets. To suppress ground clutter effectively in LSS target detection, a robust transmit beamforming algorithm has been proposed in this paper. Sidelobes in the ground side can be cut down, with the excess energy concentrated on the air side, which would be cleaner and simpler. The objective function is a second-order cone programming problem and can be solved by the convex optimization algorithm. With the consideration of taking full advantage of transmit power, the weight vector is further processed under the unimodular constraint. Numerical experiments are carried out to demonstrate the validity and superiority of the proposed method.

## 1. Introduction

Noncooperative low-altitude slow-speed small (LSS) targets refer to targets with flying height no more than 1000 meters, flying speed less than 200 kilometres per hour, and radar cross section (RCS) not more than 2 square meters [1, 2]. LSS targets include unmanned aerial vehicles (UAVs), birds, kites, light and super airplanes, and gliders. Owing to low cost, high flexibility, and simple operation, LSS targets, such as UAVs and micro aircrafts, have been widely utilized in many application scenarios, posing great threats to public security and personal privacy [3, 4]. LSS targets often move in complex low-altitude areas with many obstructions. On the other hand, due to the small RCS of the LSS target, the radar echo is weak. In addition, LSS targets fly at slow speeds, resulting in insignificant Doppler frequency [5]. Therefore, it is extremely difficult for the detection, localization, tracking, and classification of LSS targets. With the gradual opening of airspace, the increasing threats of LSS targets have motivated researchers to investigate LSS targets surveillance systems.

Generally speaking, the technologies utilized for LSS targets surveillance mainly include acoustic-based, video-based, radio-frequency (RF)-based, and radar-based technologies [6]. The acoustic signatures of drone-like micro aircrafts can be obtained via analysis in both the time and frequency domains. Shi et al. [7] built an acoustic-based surveillance system, in which a detection fusion algorithm and a new time delay of arrival estimation algorithm based on the Bayesian filter are applied to improve the performance of drone detection and localization. However, the sounds are generated by the motors or fast rotating propellers. Therefore, the acoustic-based surveillance system is not suitable for birds or kites monitoring. An object can be detected using its appearance features [8] or/and its motion features cross-consecutive frames [9]. For instance, a novel spatiotemporal saliency method (NSTSM) was proposed in [10] for LSS infrared target detection. NSTSM uses the motion information of target pixels and background pixels in forward and backward frames to further suppress background clutter. Wang et al. [11] utilized a relocalization framework to address the problem of small flying object tracking through computer vision. Nevertheless, the performances of video-based methods would decline because of occlusion or bad weather. A real-time passive coherent location system based on digital video broadcast has been proposed in [12], in which the detailed demonstration of the hardware system, signal processing, and field experiment is presented. RF-based surveillance approaches make use of the specific communication frequency bands, whereas this kind of method faces severe challenges due to preset flight path, ambient RF noise, and multipath effect.

Compared to acoustic-based, video-based, and RF-based methods, radar technology with its all-weather capability can play an important role in LSS targets detection. W-band radar was used to make a substantial contribution to avoid the growing threats from LSS aerial vehicles [13]. A small-scale digital array radar prototype, operating in the S band, was developed to detect a slow-moving micro-UAV target at a relatively long range [14]. A decoupled directional range indication scheme based on coprime FDA was proposed in [15]. A larger array aperture and a higher degree of freedom can be achieved so that the presented framework could locate the direction and distance of the target without coupling and form a thumbtack-shaped beampattern. Hough transform was used to improve the performance of general high-resolution radar in detecting and tracking UAVs [16]. A coherent integration method based on stretch processing and chirp-z transform in the frequency domain is proposed for passive bistatic radar to improve UAV detection performance [17].

Resisting the strong ground clutter in echoes can raise the input signal-to-clutter ratio (SCR) for radar receivers directly, so as to improve the LSS target detection performance, which has not been mentioned in the literature. As a result, beampatterns can be designed to provide a higher detection performance [18–22]. Considering that the background interference of high-altitude targets is relatively simple and clean, while the low-altitude background has much more complex background interference. In this paper, a robust transmit beamforming algorithm has been proposed to suppress the ground clutter for LSS target detection. The weight vector has been optimized to suppress sidelobes in the direction of the ground and interferences while maintaining the mainlobe constant. The objective function can be converted to a second-order cone programming (SOCP) problem and solved by well-established interior-point methods (IPM). Then, with the consideration of exploiting the transmit powerfully, amplitude normalization is employed to make the weight vector unimodular. Numerical experiments were implemented to verify the effectiveness of the proposed approach.

## 2. Signal Model

Consider a uniform linear array (ULA) with *N* array elements separated from each other by a distance *d*. The transmit signal of the nth-array at t-time can be expressed as

(1) $$\begin{array}{c} x_{n}\left(t\right)=s_{n}\left(t\right)e^{j2\pi f_{0}t},\;n=1,2,3,\ldots ,N, \end{array}$$

where *s*_*n*_(*t*) represents the baseband signal and *f*_0_ denotes the carrier frequency. After decomposed into amplitude and phase, the baseband signal *s*_*n*_(*t*) is presented as

(2) $$\begin{array}{c} s_{n}\left(t\right)=\alpha_{n}\left(t\right)e^{j\varphi_{n}\left(t\right)}. \end{array}$$

Assuming that the distance and azimuth of a far-field target to the reference array are *r* and *θ*, respectively, then the transmitted signal propagated to the target can be expressed as

(3) $$\begin{array}{c} \frac{1}{r_{n}}\omega_{n}s_{n}\left(t-\tau_{n}\right)e^{j2\pi f_{0}\left(t-\tau_{n}\right)}=\frac{1}{r_{n}}\omega_{n}x_{n}\left(t-\tau_{n}\right), \end{array}$$

where 1/*r*_*n*_ represents the path attenuation factor and *ω*_*n*_ denotes the weight coefficient for the transmitter. Since it is assumed that the differences in path attenuation factors for individual arrays in the far-field situation can be negligible, 1/*r*_*n*_ is considered to be equal to 1/*r*_*n*_ approximately for each transmitter antenna. *τ*_*n*_ represents the propagation time of the nth-array relative to the reference array to the objective and can be written as

(4) $$\begin{array}{c} \tau_{n}=\frac{r+\left(n-1\right)d\;\sin\theta }{c}. \end{array}$$

In the narrowband case, the baseband signal envelope changes slowly over time; therefore, we can get *s*_*n*_(*t* − *τ*_*n*_) ≈ *s*_*n*_(*t*). Then, the signal emitted to the target can be further expressed as

(5) $$\begin{array}{c} \frac{1}{r_{n}}\omega_{n}x_{n}\left(t-\tau_{n}\right)\\ \approx \frac{1}{r}\omega_{n}\alpha_{n}\left(t\right)e^{j\varphi_{n}\left(t\right)}e^{j2\pi f_{0}\left(t-\left(r+\left(n-1\right)d\;\sin\theta /c\right)\right)},\\ =\frac{1}{r}e^{j2\pi f_{0}\left(t-\left(r/c\right)\right)}\omega_{n}s_{n}\left(t\right)e^{-j2\pi \left(\left(n-1\right)d\;\sin\theta /\lambda \right)}, \end{array}$$

where *λ* is the carrier wavelength. Suppose that each array emits the same baseband signal, thus *s*_*n*_(*t*) is equal to *s*(*t*), the sum of transmitted signals of the ULA array at the direction *θ* that can be expressed as

(6) $$\begin{array}{c} y\left(t\right)=\sum_{n=1}^{N}\frac{1}{r_{n}}\omega_{n}x_{n}\left(t-\tau_{n}\right),\\ \approx \frac{1}{r}e^{j2\pi f_{0}\left(t-\left(r/c\right)\right)}s\left(t\right)\sum_{n=1}^{N}\omega_{n}e^{-j2\pi \left(\left(n-1\right)d\;\sin\theta /\lambda \right)},\\ =\frac{1}{r}e^{j2\pi f_{0}\left(t-\left(r/c\right)\right)}s\left(t\right)\cdot \omega^{H}a\left(\theta \right), \end{array}$$

where

(7) $$\begin{array}{c} \omega ={\left[\omega_{1},\omega_{2},\ldots ,\omega_{N}\right]}^{T},\\ a\left(\theta \right)={\left[1,e^{-j2\pi \;d\;\sin\theta /\lambda },\ldots ,e^{-j2\pi \left(N-1\right)d\;\sin\theta /\lambda }\right]}^{T}, \end{array}$$

are the weight vector of the array and transmit steering vector at *θ*, respectively.

## 3. Proposed Method

As LSS target detection suffers from severe ground clutter and other slow small jammers at low altitudes, the echo power reflected from the ground should be as low as possible. Let Θ_*G*_ represent the set of locations in the ground side, the power constraint in transmit beamformer can be written as

(8) $$\begin{array}{c} {\left|\omega^{H}a\left(\theta \right)\right|}^{2}\leq \delta ,\;\forall \theta \in \Theta_{G}, \end{array}$$

where *δ* is the prescribed sidelobe peak value for locations in Θ_*G*_ and can be specified to different values for different locations according to actual requirements.

Actually, the errors in array antenna spacing, channel amplitude, and channel phase would lead to distortion of beamforming, which will reduce the spatial filtering capability as well as the robustness of the transmit beampattern.

Assuming that the ideal position of the *n*th array element is *p*_*n*_, the exact position of the *n*th element is

(9) $$\begin{array}{c} {\hat{p}}_{n}=p_{n}+\Delta p_{n}, \end{array}$$

where Δ*p*_*n*_ denotes the position error of the *n*th transmit antenna.

The ideal weight vector of the beamformer is given in (7). Suppose that the *n*th weighting coefficient can be written as

(10) $$\begin{array}{c} \omega_{n}=g_{n}e^{j\phi_{n}}, \end{array}$$

where *g*_*n*_ and *ϕ*_*n*_ are the ideal amplitude and phase weighting factors, respectively. Due to the channel error in practical engineering, the actual amplitude and phase weighting coefficients are

(11) $$\begin{array}{c} {\hat{g}}_{n}=g_{n}+\Delta g_{n},\\ {\hat{\phi }}_{n}=\phi_{n}+\Delta \phi_{n}, \end{array}$$

where Δ*g*_*n*_ and Δ*ϕ*_*n*_ represents the amplitude error and phase error of the *n*th weighting coefficient, respectively.

Assume that Δ*g*_*n*_, Δ*ϕ*_*n*_, and Δ*p*_*n*_(*n*=1,2,…, *N*) are all statistically independent and random variables, obeying the zero-mean Gaussian distribution. The variances of Δ*g*_*n*_, Δ*ϕ*_*n*_, and Δ*p*_*n*_ are *σ*_*g*_^2^, *σ*_*ϕ*_^2^, and *σ*_*p*_^2^, respectively. Define *σ*_*λ*_=(2*π*/*λ*) · *σ*_*p*_, the practical response of the beampattern can be represented as

(12) $$\begin{array}{c} \hat{F}\left(\theta \right)={\left|{\hat{\omega }}^{H}\hat{a}\left(\theta \right)\right|}^{2},\\ ={\left|\sum_{n=1}^{N}{\hat{g}}_{n}e^{\left(j\left({\hat{\phi }}_{n}-2\pi {\hat{p}}_{n}\sin\left(\theta \right)/\lambda \right)\right)}\right|}^{2}, \end{array}$$

where $\hat{\omega }$ and $\hat{a}\left(\theta \right)$ are the actual weight vector and array steering vector, respectively. When all the above errors are tiny, the amplitude expect of the actual beam response is

(13) $$\begin{array}{c} E\left\{\hat{F}\left(\theta \right)\right\}=F\left(\theta \right)e^{-\left(\sigma_{\phi }^{2}+\sigma_{\lambda }^{2}\right)}+\sum_{n=1}^{N}g_{n}^{2}\left(\sigma_{\phi }^{2}+\sigma_{\lambda }^{2}+\sigma_{g}^{2}\right), \end{array}$$

where *F*(*θ*) is the ideal beampattern. The sensitivity function is expressed as

(14) $$\begin{array}{c} T_{se}=\sum_{n=1}^{N}g_{n}^{2}={\left\|\omega \right\|}_{2}^{2}. \end{array}$$

The first part in (15) is the ideal beampattern multiplied by an attenuation factor, which affects the overall size of the beamforming in each angular grid, and does not affect the beam gain. The second part in (15) is the product of the sum of error variances with *T*_*se*_ in (16), which influences the sidelobes of the beampattern. It can be found that with constant error variances, the smaller the *T*_*se*_, the higher the robustness of beamforming.

To improve LSS target detection performance robustly, the transmit beampattern should be optimized following 4 principles. (1) The *ℓ*_2_ norm of the weight vector should be minimized to ensure the robustness. (2) The response at mainlobe should be constant, while nulls should be placed in the locations with strong interferences. (3) The sidelobes oriented to the ground should be lower than a threshold. (4) The sidelobe level growth in the air side cannot be too significant. In this way, the weight vector optimizing problem can be formulated as follows:

(15) $$\begin{array}{c} \underset{\omega }{\min}{\left\|\omega \right\|}^{2}\\ \text{s.t. }\omega^{H}a\left(\theta_{0}\right)=1\\ {\left|\omega^{H}a\left(\theta_{s}\right)\right|}^{2}\leq \delta_{s},\;\forall \theta_{s}\in \Theta_{S},\\ {\left|\omega^{H}a\left(\theta_{a}\right)\right|}^{2}\leq \delta_{a},\;\forall \theta_{a}\in \Theta_{A}, \end{array}$$

where *θ*_0_ is the mainlobe location, while *θ*_*s*_ represents the location with interference or in the ground side. *θ*,_*a*_ denotes the location in the air side. Θ_*S*_ and Θ_*A*_ are the sets of locations with interferences as well as those in Θ_*G*_ and in the air side, respectively. Both *δ*_*s*_ and *δ*_*a*_ are the thresholds specified according to the practical application.

The problem in (17) can be converted to a SOCP problem:

(16) $$\begin{array}{c} \underset{\omega }{\min}{\left\|\omega \right\|}^{2}\\ \text{s.t. }\omega^{H}a\left(\theta_{\text{0}}\right)=1\\ \left|\omega^{H}a\left(\theta_{s}\right)\right|\leq \sqrt{\delta_{s}},\;\forall \theta_{s}\in \Theta_{S},\\ \left|\omega^{H}a\left(\theta_{a}\right)\right|\leq \sqrt{\delta_{a}},\;\forall \theta_{a}\in \Theta_{A}, \end{array}$$

which is a subclass of convex programming problems. SOCP problem (18) can be solved efficiently in polynomial time using IPM [23]. There are many well-constructed MATLAB toolboxes, such as CVX [24, 25] and SeDuMi [26], which can be utilized to solve SOCP problems. Here, we use CVX to find the optimal solution, which is denoted by *ω*_SOCP_.

However, the transmit signals weighted in both amplitude and phase would cause the loss of transmit power. In order to make full use of transmit power, the weight vector should be unimodular. Here, the amplitude normalization of *ω*_SOCP_ is adopted to obtain the optimal weight vector; that is,

(17) $$\begin{array}{c} \omega_{\text{opt}}=e^{j*\arg\left(\omega_{\text{SOCP}}\right)}. \end{array}$$

## 4. Simulations and Analysis

In this section, 4 simulation cases are carried out to illustrate the effectiveness and superiority of the presented approach by considering beampattern and SCR performance. In all cases, we assume that the transmit array is equipped with *N*=32 antennas with half-wavelength spacing between adjacent elements. The point target is located at an angle *θ*_0_=^0°^, which would be the angle direction of the peak mainlobe of the transmit beam. The angular pattern covers [−90°, 90°] with a mesh grid size of 0.1°. The ground side includes the locations in the range of [−90°, −5°], while the air side ranges from 5° to 90°.

**Case 1 .**

Assume that all the sidelobes in the ground side should be lower than -30 dB with sidelobes no more than −10 dB.  Figure 1 gives beampattern comparisons of the static weight vector *ω*_0_=**a**^*H*^(*θ*_0_), *ω*_SOCP_, and *ω*_opt_, respectively. It can be found that beampatterns obtained by both *ω*_SOCP_ and *ω*_opt_ have lower sidelobes in the range of [−90°, −5°] than the static beampattern *ω*_0_, while the sidelobes in the air side rang rise a little. The peak sidelobe levels in the air side of the beam formed by *ω*_0_, *ω*_SOCP_, and *ω*_opt_ are −13.24 dB, −13.17 dB, and −9.93 dB, respectively. Compared to the beam got by *ω*_0_, the sidelobe growth brought by *ω*_SOCP_ and *ω*_opt_ is 0.07 dB and 3.31 dB, respectively. As there is little interference or clutter in the air side, the sidelobe growth is acceptable. It can be found that the sidelobes in the ground side formed by *ω*_SOCP_ are lower and flatter than those obtained by *ω*_opt_. Moreover, the sidelobe growth in the air side obtained by *ω*_SOCP_ is lower than that obtained by *ω*_opt_. However, beamforming by *ω*_SOCP_ performs both amplitude and phase weighting, which would lead to transmit power loss. *ω*_opt_ performs only phase weighting, which can make full use of transmit power. The value of *ω*_0_, *ω*_SOCP_, and *ω*_opt_ can be found in Table 1.

**Case 2 .**

The suppression thresholds for sidelobes in both ground and air sides are sets according to Case 1. Directions of departure of two interferences are −20° and 35°. The threshold for interference suppression is set to −80 dB.  Figure 2 illustrates the beampatterns formed by *ω*_0_, *ω*_SOCP_, and *ω*_opt_, respectively. The detailed information about position and depth for interferences is shown in Table 2. Obviously, in contrast to *ω*_0_, both *ω*_SOCP_ and *ω*_opt_ can form nulls in interference points effectively while suppressing sidelobes in the ground side. Therefore, the proposed method can reduce the ground clutter in radar echoes as well as place nulls in interference locations. The sidelobe growth brought by *ω*_SOCP_ and *ω*_opt_ relative to *ω*_0_ is 0.12 dB and 3.37 dB, respectively. Hence, the proposed method achieves a better tradeoff between interference suppression and full use of transmit power with little sidelobe increase in the air side. The value of *ω*_0_, *ω*_SOCP_, and *ω*_opt_ in this case can be found in Table 3.

**Case 3 .**

The sidelobe thresholds for ground side are set to −20 dB, −25 dB, −30 dB, and −35 dB, respectively. Other settings are the same as those in Case 1.  Figure 3 shows the beampatterns obtained by *ω*_opt_ for different thresholds. It can be seen that the proposed method can almost meet the sidelobe suppression requirements for −20 dB, −25 dB, and −30 dB. For the −35 dB suppression requirement, only the sidelobes near the mainlobe can be reduced to −35 dB approximately. But the sidelobes in the range of [−90°, −35°] cannot be cut down effectively. The value of *ω*_opt_ for different thresholds for sidelobe suppression in the ground side is shown in Table 4.

**Case 4 .**

In this experiment, the performance of the ground clutter suppression would be analysed in view of SCR improvements in echoes. Without loss of generality, we suppose that there is no interference. Assume that the power of the target is *σ*_s_^2^, while the average power of ground clutter in each location of the ground side is *σ*_c_^2^. Therefore, SCR in the target scene can be expressed as

(18) $$\begin{array}{c} {\text{SCR}}_{i}=\frac{\sigma_{s}^{2}}{L_{g}\sigma_{c}^{2}}, \end{array}$$

where *L*_*g*_ is the number of locations in the ground side. After beamforming, the SCR of the reflection signal is

(19) $$\begin{array}{c} {\text{SCR}}_{r}=\frac{\sigma_{s}^{2}{\left|\omega^{H}a\left(\theta_{0}\right)\right|}^{2}}{\sigma_{c}^{2}\sum_{\Theta_{G}}{\left|\omega^{H}a\left(\theta \right)\right|}^{2}}\\ =L_{g}{\text{SCR}}_{i}\frac{{\left|\omega^{H}a\left(\theta_{0}\right)\right|}^{2}}{\sum_{\Theta_{G}}{\left|\omega^{H}a\left(\theta \right)\right|}^{2}}. \end{array}$$

Define the SCR improvement ratio as

(20) $$\begin{array}{c} \gamma =\frac{{\text{SCR}}_{r}}{{\text{SCR}}_{i}}\\ =L_{\text{g}}\frac{{\left|\omega^{H}a\left(\theta_{\text{0}}\right)\right|}^{2}}{\sum_{\Theta_{G}}{\left|\omega^{H}a\left(\theta \right)\right|}^{2}}. \end{array}$$

The SCR improvement ratio *γ* denotes the performance of ground clutter suppression.  Figure 4 shows the SCR improvements ratio against different threshold values for sidelobe suppression obtained by *ω*_opt_ and *ω*_0_. We can find that compared to static beamformer weight vector, the proposed method can obtain better suppression performance for ground clutter. With the suppression requirement growing strictly, the SCR improvement ratio of the proposed method declines slightly.

## 5. Conclusion

In this paper, a robust transmit beamforming approach is deduced specifically to handle with LSS targets detection problem. We have shown that by suppressing the energy of the sidelobe emitted to the ground, and irradiating the excess capacity into the clean air, the echoes from the ground reflection can be reduced greatly. So that the performance of LSS target detection can be enhanced with SCR in echoes improved. Considering the full use of transmitting power, the unimodular constraint is also implemented on the weight vector design, with a little sidelobe suppression performance declining. In our future work, how to meet the strict sidelobe suppression requirement would be studied.

## Figures and Tables

**Figure 1:** Comparisons of beampatterns formed by weight vectors *ω*_0_, *ω*_SOCP_, and *ω*_opt_.

**Figure 2:** Comparisons of beampatterns formed by *ω*_0_, *ω*_SOCP_, and *ω*_opt_ with 2 interference points in Case 2.

**Figure 3:** Beampattern comparison for different suppression requirements in Case 3.

**Figure 4:** SCR improvement comparisons against different suppression requirements.

**Table 1:** The value of *ω*_0_, *ω*_SOCP_, and *ω*_opt_ in Case 1.

*ω*_0_	*ω*_SOCP_	*ω*_opt_
1	0.0207 + 0.0156i	0.7996 + 0.6006i
1	0.0207 + 0.0054i	0.9677 + 0.2523i
1	0.0234 + 0.0011i	0.9989 + 0.0473i
1	0.0252–0.0014i	0.9986–0.0536i
1	0.027–0.003i	0.9938–0.1114i
1	0.0286–0.0042i	0.9893–0.1457i
1	0.0302–0.0049i	0.9869–0.1611i
1	0.0317–0.0054i	0.986–0.1667i
1	0.0331–0.0054i	0.9868–0.1617i
1	0.0344–0.0053i	0.9884–0.1517i
1	0.0356–0.0048i	0.9908–0.1351i
1	0.0366–0.0043i	0.9932–0.116i
1	0.0375–0.0035i	0.9957–0.0925i
1	0.0381–0.0026i	0.9977–0.0682i
1	0.0386–0.0016i	0.9992–0.041i
1	0.0388–0.0006i	0.9999–0.0142i
1	0.0388 + 0.0006i	0.9999 + 0.0142i
1	0.0386 + 0.0016i	0.9992 + 0.041i
1	0.0381 + 0.0026i	0.9977 + 0.0682i
1	0.0375 + 0.0035i	0.9957 + 0.0925i
1	0.0366 + 0.0043i	0.9932 + 0.116i
1	0.0356 + 0.0048i	0.9908 + 0.1351i
1	0.0344 + 0.0053i	0.9884 + 0.1517i
1	0.0331 + 0.0054i	0.9868 + 0.1617i
1	0.0317 + 0.0054i	0.986 + 0.1667i
1	0.0302 + 0.0049i	0.9869 + 0.1611i
1	0.0286 + 0.0042i	0.9893 + 0.1457i
1	0.027 + 0.003i	0.9938 + 0.1114i
1	0.0252 + 0.0014i	0.9986 + 0.0536i
1	0.0234–0.0011i	0.9989–0.0473i
1	0.0207–0.0054i	0.9677–0.2523i
1	0.0207–0.0156i	0.7996–0.6006i

**Table 2:** The position and depth of nulls for interferences in Case 2.

	Weight vector	*ω*_0_	*ω*_SOCP_	*ω*_opt_
−20°	Position (°)	−22	−20	−20.8
	Depth (dB)	−59	−72	−57
35°	Position (°)	34.2	35	35.3
	Depth (dB)	−61	−73	−56

**Table 3:** The value of *ω*_0_, *ω*_SOCP_, and *ω*_opt_ in Case 2.

*ω*_0_	*ω*_SOCP_	*ω*_opt_
1	0.0197 + 0.0165i	0.768 + 0.6404i
1	0.0204 + 0.0048i	0.9733 + 0.2296i
1	0.0236 + 0.0008i	0.9994 + 0.0359i
1	0.0261–0.0013i	0.9988–0.0495i
1	0.0274–0.0025i	0.9958–0.0915i
1	0.0283–0.0036i	0.9919–0.1274i
1	0.0296–0.0046i	0.988–0.1543i
1	0.0314–0.0058i	0.9832–0.1826i
1	0.0332–0.006i	0.9839–0.1787i
1	0.0349–0.0054i	0.9884–0.1517i
1	0.0362–0.0044i	0.9928–0.12i
1	0.0366–0.0038i	0.9945–0.1044i
1	0.0369–0.0032i	0.9962–0.0873i
1	0.0377–0.0028i	0.9972–0.0749i
1	0.0387–0.0022i	0.9984–0.0559i
1	0.0393–0.0009i	0.9997–0.024i
1	0.0393 + 0.0009i	0.9997 + 0.024i
1	0.0387 + 0.0022i	0.9984 + 0.0559i
1	0.0377 + 0.0028i	0.9972 + 0.0749i
1	0.0369 + 0.0032i	0.9962 + 0.0873i
1	0.0366 + 0.0038i	0.9945 + 0.1044i
1	0.0362 + 0.0044i	0.9928 + 0.12i
1	0.0349 + 0.0054i	0.9884 + 0.1517i
1	0.0332 + 0.006i	0.9839 + 0.1787i
1	0.0314 + 0.0058i	0.9832 + 0.1826i
1	0.0296 + 0.0046i	0.988 + 0.1543i
1	0.0283 + 0.0036i	0.9919 + 0.1274i
1	0.0274 + 0.0025i	0.9958 + 0.0915i
1	0.0261 + 0.0013i	0.9988 + 0.0495i
1	0.0236–0.0008i	0.9994–0.0359i
1	0.0204–0.0048i	0.9733–0.2296i
1	0.0197–0.0165i	0.768–0.6404i

**Table 4:** The value of *ω*_opt_ for different thresholds for sidelobe suppression in the ground side in Case 3.

-20 dB	−25 dB	−30 dB	−35 dB
0.9996 + 0.0281i	0.9763 + 0.2162i	0.8081 + 0.5891i	0.5435 + 0.8394i
0.996–0.0897i	0.9994 + 0.0334i	0.9943 + 0.1063i	0.9831 + 0.1831i
0.9775–0.211i	0.981–0.1938i	0.9853–0.1711i	0.992–0.126i
0.9438–0.3306i	0.9248–0.3804i	0.9341–0.357i	0.9449–0.3274i
0.8963–0.4434i	0.8646–0.5025i	0.8706–0.4919i	0.8607–0.5092i
0.8383–0.5453i	0.8104–0.5859i	0.8015–0.598i	0.7933–0.6089i
0.7729–0.6345i	0.7552–0.6555i	0.7271–0.6866i	0.6915–0.7224i
0.7028–0.7114i	0.6924–0.7216i	0.6524–0.7579i	0.622–0.783i
0.6291–0.7773i	0.6213–0.7836i	0.5707–0.8212i	0.5175–0.8557i
0.5517–0.8341i	0.5448–0.8386i	0.4902–0.8716i	0.4472–0.8944i
0.469–0.8832i	0.4636–0.886i	0.4006–0.9162i	0.3427–0.9394i
0.3794–0.9252i	0.375–0.927i	0.3132–0.9497i	0.2717–0.9624i
0.281–0.9597i	0.2757–0.9613i	0.2159–0.9764i	0.1679–0.9858i
0.1729–0.9849i	0.1657–0.9862i	0.1223–0.9925i	0.0964–0.9953i
0.0561–0.9984i	0.049–0.9988i	0.0196–0.9998i	−0.0065-i
−0.0664–0.9978i	−0.0694–0.9976i	−0.0766–0.9971i	−0.0776–0.997i
−0.1897–0.9819i	−0.1867–0.9824i	−0.1796–0.9837i	−0.1786–0.9839i
−0.3083–0.9513i	−0.3015–0.9535i	−0.2734–0.9619i	−0.2482–0.9687i
−0.4178–0.9085i	−0.4111–0.9116i	−0.3708–0.9287i	−0.3464–0.9381i
−0.5159–0.8567i	−0.5111–0.8595i	−0.4572–0.8894i	−0.4131–0.9107i
−0.6023–0.7983i	−0.5985–0.8011i	−0.5445–0.8388i	−0.5076–0.8616i
−0.6783–0.7348i	−0.6738–0.7389i	−0.6205–0.7842i	−0.5705–0.8213i
−0.7457–0.6663i	−0.7402–0.6724i	−0.6958–0.7182i	−0.6601–0.7512i
−0.8062–0.5917i	−0.8002–0.5997i	−0.7608–0.649i	−0.7181–0.6959i
−0.8607–0.5092i	−0.8531–0.5217i	−0.8237–0.567i	−0.8008–0.599i
−0.9089–0.417i	−0.8971–0.4418i	−0.8778–0.479i	−0.8525–0.5226i
−0.9494–0.3141i	−0.9328–0.3604i	−0.9272–0.3744i	−0.9221–0.387i
−0.9796–0.2007i	−0.964–0.266i	−0.9671–0.2542i	−0.9619–0.2734i
−0.9968–0.0796i	−0.9912–0.1326i	−0.9942–0.1076i	−0.9971–0.0762i
−0.999 + 0.0447i	−0.9981 + 0.0622i	−0.9964 + 0.0852i	−0.9914 + 0.1305i
−0.986 + 0.1666i	−0.9581 + 0.2866i	−0.9346 + 0.3558i	−0.9042 + 0.4272i
−0.9596 + 0.2815i	−0.8892 + 0.4575i	−0.6316 + 0.7753i	−0.312 + 0.9501i

## Data Availability

No dataset were used in this paper. The simulation data will be made available from the corresponding author upon request.

## Abbreviations

(*g*)^*T*^ and (*g*)^*H*^: The operations of transpose and conjugate transpose, respectively
‖*g*‖_2_: The Euclidean *ℓ*_2_ norm
*e* ^(*g*)^: The exponential operator
arg(*g*): An operator to get the phase of the parameter in radian
*e*: The Hadamard product
$j=\sqrt{-1}$: The imaginary unit.
